# Expediting support for the pregnant mothers to obtain antenatal care at public health facilities in rural areas of Balochistan province, Pakistan

**DOI:** 10.12669/pjms.313.7082

**Published:** 2015

**Authors:** Abdul Ghaffar, Sathirakorn Pongpanich, Najma Ghaffar, Robert Sedgwick Chapman, Sheh Mureed

**Affiliations:** 1 Dr. Abdul Ghaffar, Planning Officer, Health Department Health Department, Government of Balochistan, Pakistan; 2 Dr. Sathirakorn Pongpanich, Associate Professor, College of Public Health Sciences, Chulalongkorn University, Bangkok, Thailand; 3 Dr. Najma Ghaffar, Associate Professor of Gynae and Obstetrics, Bolan Medical College, Pakistan; 4 Dr. Robert Sedgwick Chapman, Lecturer, College of Public Health Sciences, Chulalongkorn University, Bangkok, Thailand; 5 Dr. Sheh Mureed, Postdocotorate Scholar, College of Public Health Sciences, Chulalongkorn University, Bangkok, Thailand

**Keywords:** Antenatal care, Maternal Health, Pregnancy, Public Health facility, Utilization

## Abstract

**Objectives:**

To identify, and compare relative importance of, factors associated with antenatal care (ANC) utilization in rural Balochistan, toward framing a policy to increase such utilization.

**Methods:**

This cross sectional study was conducted among 513 pregnant women in Jhal Magsi District, Balochistan, in 2011. A standardized interviewer-administered questionnaire was used. Predisposing, enabling, and reinforcing factors were evaluated with generalized linear models (Poisson distribution and log link).

**Results:**

Prevalence of any ANC was only 14.4%. Predisposing, enabling, and reinforcing factors were all important determinants of ANC utilization. Reinforcing factors were clearly most important, husband’s support for ANC was more important than support from other community members. Among predisposing factors, higher income, education, occupation, and better knowledge regarding benefits of ANC were positively and statistically significantly associated with ANC However increased number of children showed negative association. Complications free pregnancy showed positive significant association with ANC at public health facility among enabling factors.

**Conclusion:**

It is very important to increase antenatal care utilization in the study area and similar areas. Policy to achieve this should focus on enhancing support from the husband.

## INTRODUCTION

Many developing countries including Pakistan are striving to reduce maternal deaths, particularly in rural and peri-urban areas.^1^ According to Pakistan demographic and health survey (PDHS) 2007, estimated nationwide maternal mortality rate (MMR) is 276/100,000 live births. In Balochistan Province the MMR is 785 deaths/100,000 live births, Antenatal Care (ANC) coverage in Pakistan is 61% for at least one visit, and is 39% for 4 or more visits. The Balochistan province district health information system (DHIS) for 2010 showed only 15% registration of the pregnant mothers for ANC at least for one visit.^2^ A healthy end of pregnancy for both fetus and mother relies on cautious care throughout pregnancy.^3^

In most parts of Balochistan province women lack both knowledge and danger signs in pregnancy and information regarding ANC at public health facilities. Many do not know how to seek care when a complication occurs during pregnancy. The attitudes and behaviors of health care providers in ANC clinics compound this problem by failing to respect the privacy, confidentiality, and traditional beliefs of the women, and may thus negatively influence the use of ANC as well as other maternal and child health (MNCH) services at large, families and communities may underestimate the importance of ANC.^4^,^5^

The local communities here in Balochistan are still living under strict social customs, educating women is often a taboo, their mobility out of home is limited without a companion male (e.g., husband or brother).^6^ This feudal situation is prone to generating conflicts whose consequences most severely affect women and children. Health system is providing doorstep maternal and child health services through different parallel programs like MNCH, Lady Health worker Program (LHW). Even so, the health system is unable to achieve targeted objectives.^7^,^8^

Therefore, the present study aimed to identify the supporting factors, grouped in predisposing, enabling and reinforcing factors that may increase obtaining of ANC services at public health facilities among pregnant women in Jhal Magsi District, Balochistan.

## METHODS

This community-based cross-sectional study was conducted in August to December 2011 at District Jhal Magsi (JM). This study focused on educational and organizational diagnosis and analysis addressed predisposing, enabling and reinforcing factors related to utilization of ANC.

The main outcome variable was routine antenatal care (at least one visit) at a government facility during the current or most recent pregnancy without major complications such as bleeding, hypertension, or eclampsia. The predisposing factors (total 7 factors) were age, education, occupation, income, parity, and knowledge and attitude about ANC. Enabling factors (total 3 factors) were travel cost, distance and minor complications during pregnancy (such as vomiting, body aches, or anemia). Reinforcing factors (total 13 factors) were favorable opinion, active encouragement, information, and financial support from husband, mother-in-law and other community members (included support from other relatives, friends and neighbors), as well as information from health care personnel and electronic media i.e. TV and radio. We believe that this model is appropriate for the study, because it allows for evaluation of the importance of male involvement (and other potentially relevant factors) in obtaining ANC.^9^

### Study samples and sampling

A three-stage sampling process was employed for participant selection. Subjects in Union Council Pattri were identified using the Expanded Program on Immunization (EPI) lists.^10^ According to the EPI list of 2011, Pattri had a total population of 17,375 and about 712 ladies became pregnant per year.

We were able to enroll 513 pregnant women, from 15 villages, this number of sample size is sufficient to detect the difference in prevalence between exposed and unexposed groups, if the prevalence in the unexposed is 10% and the prevalence in exposed group is 20% and there are twice as many people exposed as unexposed, with 95% confidence and 80% power.

### Data Analysis

Descriptive statistics were used to characterize sociodemographic characteristics of the respondents, data were analyzed in four steps, using multiple regression models; final model was constructed, which included only independent variables for which p<0.2 in the step 3 model.

Data were analyzed with generalized linear models with distribution=Poisson and link=log. Relative importance of predisposing, enabling, and reinforcing characteristics was assessed by comparing quasi-likelihoods (QLs) for models in which each type of characteristic was dropped out of the final step 4 model described above.^11^ In all analyses p-values<0.05 were considered statistically significant. Data were analyzed using the Statistical Package for Social Sciences (SPSS) for Windows, version 16.

The Ethics Review Committee for Research Involving Human Research Subjects, Health Sciences Group, Chulalongkorn University, Bangkok, Thailand, granted ethical approval, vide letter no COA No. 14312011for this study in 2011. Permission to conduct research in the District Jhal Magsi was also obtained from the District Health officer and provincial Secretary Health Department, Government of Balochistan.

## RESULTS

### Demographic and descriptive statistics

Mean age of the pregnant ladies in the study was 24.7 ± 4.1 years, and number of Children born mean was 4.9 ± 1.8, mean distance from the nearest health facility providing ANC services was 17.7 km ± 10.4, and mean family income was 6548.7 ± 3743 Pakistan rupees ($90 US). Most (98.1%) of the study participants were housewives and 7.8% had any formal education. 74 (14.4%) had visited a public health facility for ANC during their last or current pregnancy without major complications. The pregnancy for which the participant reported ANC history was not specified. Among these 74 women, 47, 22, and 5 made ANC visits in all 3 trimesters, only two trimesters, and only one trimester, respectively.

Table-I shows association of predisposing factors with ANC, formal education, family income, occupation and knowledge about ANC showed positive association however No. of Children born showed negative association.

**Table-I:** Associations of predisposing factors with obtaining any antenatal care at a public health facility (step 2 model for predisposing factors).

Predisposing Factors	Coefficient	Std. Error	Relative Risk	95%CI		P-value
				Lower	Upper	
Any formal education	0.36	0.234	1.43	0.90	2.27	0.125
Occupation as government servant vs. other occupations	0.28	0.182	1.32	0.92	1.89	0.126
Higher family income (≥$90 US per month)	0.94	0.279	2.55	1.48	4.41	0.001
≥ 4 vs. <4 children born alive	-0.99	0.301	0.37	0.21	0.67	0.001
Higher knowledge about ANC & its benefits	2.48	0.252	11.94	7.29	19.56	<0.001
Intercept	-1.48	0.538				0.006

Table-II shows associations of enabling factors with obtaining ANC. In comparison to a distance of <16 km, a distance of 16-20 km was positively associated with ANC, and a longer distance was negatively associated. Lower travel cost and absence of minor complications during pregnancy were positively and significantly associated with ANC utilization.

**Table-II:** Associations of enabling factors with obtaining any antenatal care at a public health facility (step 2 model for enabling factors).

Enabling Factors	Coefficient	Std. Error	Relative Risk	95%CI		P-value
				Lower	Upper	
Distance (km) to public antenatal care facility						
≤15			1			
16-20	0.46	0.103	1.59	1.30	1.94	<0.001
21-30	-0.84	0.599	0.43	0.13	1.39	0.160
Lower vs. higher travel cost to public health facility	1.24	0.135	3.47	2.66	4.52	<0.001
No minor complications during pregnancy	2.36	0.308	10.65	5.83	19.48	<0.001
Intercept	-4.085	0.341				<0.001

Table-III shows associations between ANC and reinforcing factors. Three dimensions out of four (except favorable opinion) from husband support were significantly associated with ANC utilization. Mother-in-law providing information and financial support showed negative association with antenatal care at public health facility. Active encouragement from other community members also showed significant positive association. Information collectively from health personnel and electronic media also showed significant positive association. The final model for all types of factors is summarized in Table-IV. This model contained 16 independent variables (5 predisposing, 3 enabling, and 8 reinforcing). In the final 16 variable model 4 predisposing factors, one enabling and 5 reinforcing factors prove to be most important factors and 3out of 4 domains of husband’s support in reinforcing factors are statistically significant Table-IV.

**Table-III:** Associations of reinforcing factors with obtaining any antenatal care at a public health facility (step 2 model for reinforcing factors).

Reinforcing Factors	Coefficient	Std. Error	Relative Risk	95%CI		P-value
				Lower	Upper	
*Support from Husband*						
Active encouragement to obtain ANC	1.58	0.347	4.85	1.98	6.37	<0.001
Providing Information to obtain ANC	2.55	0.357	12.89	6.41	25.95	<0.001
Financial support for ANC	1.49	0.762	4.44	0.99	19.78	0.051
*Support from Mother-in-law*						
Active encouragement to obtain ANC	0.27	0.172	1.31	0.99	1.72	0.05
Providing Information to obtain ANC	-0.41	0.189	0.66	0.47	0.93	0.01
Financial support for ANC	-0.24	0.096	0.78	0.64	0.94	0.01
*Support of other community members*						
Active encouragement to obtain ANC	0.33	0.178	1.40	0.98	1.98	0.06
*Information regarding ANC*						
From Health Personnel and electronic media	1.59	0.303	4.92	2.71	8.91	<0.001
Intercept	-5.72	0.985				<0.001

**Table-IV:** Joint associations of predisposing, enabling, and reinforcing factors with obtaining any antenatal care at a public health facility (from final step 4 model).

Factor	Coefficient	Std. Error	Relative Risk	95%CI		P-value
				Lower	Upper	
*Predisposing Factors*						
Any formal education	0.39	0.106	1.48	1.20	1.82	<0.001
Higher family income (≥90 US $ per month)	0.57	0.091	1.77	1.48	2.12	<0.001
≥ 4 vs. <4 children born alive	-0.42	0.147	0.65	0.49	0.87	0.004
Higher knowledge about ANC & its benefits	0.74	0.153	2.10	1.56	2.84	<0.001
*Enabling Factors*						
No minor complications during pregnancy	0.87	0.134	2.40	1.85	3.13	<0.001
*Reinforcing Factors*						
Information regarding ANC from Health Personnel and electronic media	0.41	0.100	1.51	1.24	1.83	<0.001
*Support from Husband*						
Active encouragement to obtain ANC	0.71	0.131	2.05	1.58	2.66	<0.001
Providing Information	0.50	0.092	1.64	1.37	1.97	<0.001
Financial support	0.89	0.179	2.44	1.72	3.47	<0.001
*Support from Mother-in-law*						
Financial support for ANC	0.29	0.076	1.35	1.16	1.56	<0.001
Intercept	-3.23	0.328				<0.001

## DISCUSSION

In rural areas of Pakistan majority of women are uneducated, have high fertility rates and rural dwellers have low income. Most of the participants in this study were also illiterate, had mean number of Children born 4.8 their mean family income was <$90 US per month. Mean distance from the public health facility and household reflects scattered population in Balochistan province.

Overall antenatal care (for at least one visit from public health facility) was low (14.4%). Data from Balochistan province DHIS for the year 2010 showed 15% registration of the pregnant mothers for ANC seeking,^2^ such a low prevalence in the province emphasizes the need for increasing utilization of ANC.

According to the results of this study reinforcing factors especially Husband’s support proved to most influential factors in terms of Information, active encouragement to obtain ANC and financial support from mother in law as well.^12^-^14^ Previous studies on the relationship between ANC and social support have yielded mixed results. Women with greater support from their husband and mother-in-law generally have an increased ability to use ANC services, particularly in South Asia.^15^-^17^ A study conducted in Nepal revealed that women educated during antenatal period with their husbands were more likely to be highly prepared for birth compared with women receiving education alone.^18^

Support from other family members like mother in law significantly affected use of ANC, Older women especially mothers-in-law did not consider ANC essential during pregnancy and often discouraged their daughters-in-law from attending ANC in rural Bangladesh.^19^,^20^ Information through health personnel and electronic media also showed positive association for obtaining ANC from public health facility as community health workers are the most reliable source for dissemination of information and knowledge related to ANC and public health facilities in the rural communities.

Association of predisposing factors like knowledge of ANC and information from health personnel in this study suggests that in rural areas community health workers can access these women and play vital role in dispensing information regarding ANC services at public health facility.^20^ Family income and education are significantly associated with antenatal care utilization, it is evident from the literature that female literacy is powerful predicator to the social development of communities and utilization of modern facilities provided by the governments.^20^

Enabling factors included were low travel cost and absence minor complications during pregnancy, however travel cost lost its significance in the final model. Studies have shown that Pakistani population prefer to utilize private health facilities more as compared to the public health sector during ailment apart of travel cost and distance.^17^

## CONCLUSION

This study showed that all three factors including predisposing, enabling and reinforcing factors were important; however reinforcing factors have strong influence on the uptake of ANC in comparison with enabling and predisposing factors. Findings of this study suggests considering support from husband is important to design effective community-based public health interventions to improve maternal health during pregnancy in rural areas in a vertically integrated Health Care System in case of Balochistan Province.
